RETRACTED

# Analysis of Clinical Characteristics and Psychoacoustic Indexes in Different TCM Syndromes of Idiopathic Tinnitus

**DOI:** 10.1155/2021/2446357

**Published:** 2021-09-25

**Authors:** Yan Niu, Jinmei Ning, Shubo Zhao, Chao Fang

**Affiliations:** ^1^Department of Otolaryngology, The Second Affiliated Hospital of Kunming Medical University, Kunming, Yunnan 650101, China; ^2^Department of Otolaryngology, The First People's Hospital of Qujing, Qujing, Yunnan 655000, China; ^3^The First Hospital of Putian, Putian, Fujian 351100, China

## Abstract

**Objective:**

To explore the differences in clinical characteristics and psychoacoustic indexes of various traditional Chinese medicine (TCM) syndromes in patients with idiopathic tinnitus.

**Methods:**

312 patients with idiopathic tinnitus in our hospital from December 2017 to March 2020 were selected; divided into the wind evil invasion group (*n* = 61), the liver fire disturbance group (*n* = 69), the phlegm fire stagnation group (*n* = 42), the spleen and stomach weakness group (*n* = 48), and the kidney essence loss group (*n* = 92) according to the medical syndrome type and the detailed medical history; and clinical characteristics of patients in each group were compared.

**Results:**

The kidney essence loss group's age and course of disease were older and longer than those of other syndrome groups, and the wind evil invasion group's disease course was shorter than the liver fire disturbance, phlegm fire stagnation, and spleen and stomach weakness groups (*P* < 0.05). The PSQI score of all patients was higher than 7 points, but there was no obvious difference between the groups (*P* > 0.05). The SAS score of the liver fire disturbance and the phlegm-fire stagnation groups was higher than that of the wind evil invasion, the spleen and stomach weakness, and the kidney essence loss groups, and the SDS score of the spleen and stomach weakness and the kidney essence loss groups was higher than that of the wind evil invasion, the liver fire disturbance, and the phlegm and fire stagnation groups (*P* < 0.05). The kidney essence loss group's total hearing loss rate (92.39%) was higher than the other syndrome groups, and the wind evil invasion group's total hearing loss rate (8.19%) was lower than the other syndrome groups (*P* < 0.05); the low to medium frequency tone of tinnitus's rate in the wind evil invasion group, liver fire disturbance group, and phlegm fire stagnation group was higher than the spleen and stomach weakness group and the kidney essence loss group, but the high frequency tone of tinnitus's rate was opposite. The tinnitus loudness in these groups was higher than the spleen and stomach weakness and kidney essence loss group (*P* < 0.05).

RETRACTED

**Conclusion:**

In addition to the wind evil invasion type, most tinnitus patients may have different levels of psychological disorders. So, in the treatment of idiopathic tinnitus, in addition to the disease itself, paying more attention to the psychological status of the patient is one better therapeutic method. Besides, clinical characteristics and the psychoacoustic indexes of patients with idiopathic tinnitus have a certain correlation with the TCM syndromes.

## 1. Introduction

Idiopathic tinnitus refers to the presence of tinnitus in the ear or head of the patient in a silent environment and can only be heard by the patient. It is the most common type of tinnitus and seriously worsens the good mood and life of the patient [1]. The pathogenesis of idiopathic tinnitus is still unclear. At present, it is generally believed that both organic factors and neurological factors can cause idiopathic tinnitus. Common organic factors include external auditory canal obstruction, otitis media, auditory nerve damage, and systemic diseases. Neurological factors include the abnormalities of neurological activity, tympanic nerve plexus reflex, visceral nerve impulse abnormalities, and psychological emotions. The main current treatment methods include drug therapy, habit therapy, and electrical stimulation [2, 3]. Among them, traditional Chinese medicine (TCM) has unique advantages in the treatment of idiopathic tinnitus due to the concept of overall and the concept of syndrome differentiation. Syndrome differentiation and treatment is the core idea of TCM, but it is often subjective, and there are many types of traditional Chinese medicines and proprietary Chinese medicines for treating idiopathic tinnitus. If the syndrome is not accurately differentiated, not only the corresponding treatment effect will not be achieved but also the condition of patients even worsened [4, 5]. Therefore, in addition to the traditional evidence of syndrome differentiation collected by subjective observation, if it can be combined with objective examination indicators and other clinical features to perform syndrome differentiation, it will be of great benefit to the accurate differentiation of symptoms and signs of idiopathic tinnitus. Based on this, this study explored the differences in clinical features and psychoacoustic indicators among the various TCM syndromes in patients with idiopathic tinnitus, in order to provide a certain reference basis for TCM syndrome differentiation and treatment.

## 2. Materials and Methods

### 2.1. General Information

A total of 312 patients with idiopathic tinnitus admitted to our hospital from December 2017 to March 2020 were selected. According to the different types of TCM syndromes, they are divided into two categories: deficiency and excess. Excess group includes wind evil invasion group (61 cases), liver-fire disturbance group (69 cases), and phlegm-fire stagnation group (42 cases). Deficiency group includes spleen and stomach weakness group (48 cases) and kidney essence loss group (92 cases). This study was approved by the ethics committee of our hospital, and the patients and family members agreed and signed an informed consent form.

RETRACTED

### 2.2. Diagnostic Criteria

#### 2.2.1. Modern Medicine Diagnostic Criteria

We refer to the “Clinical Practice Guideline: Tinnitus” [6] for the classification and diagnostic criteria of idiopathic tinnitus. The patient has tinnitus which is continuous or intermittent, in the ear or skull due to unknown reasons, and the duration exceeds 1 min, which may be accompanied by hearing impairment or not, adverse psychological reactions, acute or chronic onset.

#### 2.2.2. TCM Diagnostic Criteria

*(1) Wind evil invasion*. Sudden tinnitus, accompanied by headache, vertigo, aversion to wind, fever, itching in the ears, red tongue with thin and white tongue coating, and floating and rapid pulse.

*(2) Liver fire disturbance*. Sudden tinnitus, in some patients, may be accompanied by deafness, headache, red face, vexation and irritability, bitter mouth, and dry throat. In case of poor mood, tinnitus symptoms will aggravate, with red tongue, yellow coating, and wiry and rapid pulse.

*(3) Phlegm-fire stagnation*. Tinnitus sounds like cicada chirping, chest stuffiness and excessive phlegm, distending pain under ears, frequent sighing, unsmooth urination and defecation, thin, yellow and greasy tongue coating, and wiry and slippery pulse.

*(4) Spleen and stomach weakness*. Tinnitus, deafness, physical and mental fatigue, loss of appetite, loose stool, aggravated symptoms when tired, relieved at rest, thready and weak pulse, and white and greasy coating.

*(5) Kidney essence loss*. Tinnitus, deafness, fever in palms and soles, dry mouth, soreness and weakness of waist and knees, flushing of both cheeks, red tongue, and thready and weak pulse.

### 2.3. Inclusion Criteria

Meeting the relevant diagnostic criteria for tinnitus; TCM syndrome type was one of wind evil invasion, liver fire disturbance, phlegm-fire stagnation, spleen and stomach weakness, and kidney essence loss; age 18∼65 years old; high compliance; cooperation with various examinations; and complete the filling of relevant scales.

### 2.4. Exclusion Criteria

Patients with objective tinnitus; cognitive dysfunction; conductive hearing loss; the TCM syndrome type does not conform; combine with heart, liver, kidney, or other system severity disease.

RETRACTED

### 2.5. Research Methods

Collect the general information of patients, including gender, age, course of disease, and side. The Pittsburgh Sleep Quality Index (PSQI), self-rating anxiety scale (SAS), and self-rating depression scale, (SDS) were used to assess the sleep quality and psychological status of patients. The total PSQI score was 21 points, with 0–7 points for normal sleep and >7 points for sleep disorder, and the higher the score was, the worse the sleep quality was. SAS/SDS both contained 20 items, with the critical values of 50 points, which could be divided into 1–4 grades. The standard score <50 points indicated that there was no anxiety/depression. 50–60 points mean mild anxiety/depression; 61–70 points mean moderate anxiety/depression; ≥70 points were classified as severe anxiety/depression.

#### 2.5.1. Pure Tone Audiometry

Professionals use the ORBITER922 audiometer from Madsen, Denmark, to test all patients' hearing thresholds at 0.25∼8 kHz frequencies. If both ears have tinnitus, use the obvious side as the test ear, 0.25∼3 kHz as the low-mid frequency, and 4∼8 kHz for high frequency. The test result ≤25 dbHL is regarded as sound hearing loss, 26∼40 dbHL means mild hearing loss, 41∼70 dbHL means moderate hearing loss, and ≥71 dbHL means severe hearing loss. The total hearing loss rate = the number of all hearing loss cases/total number of cases × 100%.

#### 2.5.2. Tinnitus Detection

Use Sichuan Weidi Digital Co., Ltd. Tinnitt TM Tinnitus Comprehensive Diagnosis and Treatment Instrument to match tinnitus tones and loudness to all patients. Tone matching uses a two-tone selection method with pure tones between 0.125 and 1.25 kHz, as well as narrow-band noise and white noise, to stimulate nontest ears for matching. Loudness matching uses the same pure tone as the tinnitus tone to stimulate the nontest ears for matching.

#### 2.5.3. Determination of the Severity of Tinnitus

The tinnitus handicap inventory (THI) score is used to determine and grade: a total score of 100 points, 0–16 points (level 1, mild), 18–36 points (level 2, mild), a score of 38 to 56 (level 3, moderate), a score of 58 to 76 (level 4, severe), and a score of 78 to 100 (level 5, catastrophic).

### 2.6. Statistical Methods

Data and statistical analyses were done in SPSS22.0 and GraphPad Prism 8.4. Data plotted in linear scale were expressed as mean ± standard deviation ($\bar{x}$ ± *s*); analysis of variance was used to compare the results of multiple groups. Counting data were analyzed by *χ*^2^ test and shown as (%). The inspection level is *α* = 0.05. *P* < 0.05 indicates the difference is statistically significant. Significance is indicated with stars: ^*∗*^*P* < 0.05;

RETRACTED

## 3. Results

### 3.1. Comparison of General Conditions of Patients with Different Syndromes

The age and course of disease in the kidney essence loss group were higher than those in the other syndrome groups, and the differences were statistically significant (*P* < 0.05). The disease course of the wind pathogen invasion group was lower than that of the liver-fire, phlegm-fire stagnation, and spleen and stomach weakness groups, and the differences were statistically significant (*P* < 0.05) as shown in Table 1.

### 3.2. Comparison of Sleep Quality, Anxiety, and Depression in Patients with Different Syndrome Types

The PSQI score of all patients was >7, but there was no significant difference between the groups (*P* > 0.05). The SAS scores in the liver-fire disturbance and phlegm-fire stagnation groups were higher than those in the wind pathogen invasion, spleen and stomach weakness, and kidney essence loss groups, and they were in a moderate anxiety state. The SDS scores in the spleen and stomach weakness and kidney essence loss groups were higher than those in the wind pathogen invasion and liver fire. In the upper disturbance and phlegm-fire stagnation groups, they are all in a moderately depressed state. The differences were statistically significant (*P* < 0.05) as shown in Figures 1(a)∼1(c).

### 3.3. Comparison of Average Hearing Threshold and Hearing Loss of Patients with Different Syndrome Types

The total hearing loss rate (92.39%) of the kidney essence loss group was higher than the other groups, and the total hearing loss rate (8.19%) of the wind evil invasion group was lower than the other groups. The differences were statistically significant (*P* < 0.05) as shown in Table 2.

### 3.4. Comparison of Tinnitus in Patients with Different Syndromes

The low-to-medium tone rate of tinnitus in the wind evil invasion, the liver fire disturbance, and phlegm-fire stagnation group was higher than that in the spleen and stomach weakness and kidney essence loss group. The high-frequency tone rate was lower than that of the spleen and stomach weak and kidney essence loss group, and the tinnitus loudness was higher than that of the spleen and stomach weakness and kidney essence loss group. The differences were statistically significant (*P* < 0.05) as shown in Table 3.

## 4. Discussion

In recent years, due to the changes in people's lifestyles and the increase in various types of noise, the incidence of tinnitus continues to rise, and the treatment is difficult, which has become one of the major problems in clinical otology. About 60% of people feel or experience tinnitus in their lifetime, and among them, idiopathic tinnitus is the most common [7–9]. At present, there are many types of TCM syndromes of tinnitus, among which wind evil invasion, disturbance of liver and fire, stagnation of phlegm and fire, weakness of spleen and stomach, and loss of kidney essence are the most common [10]. Studies have reported that the onset of tinnitus is closely related to psychological factors [11, 12]. Psychotherapy is also an important measure for the treatment of tinnitus, so the clinical characteristics of the various TCM syndromes of patients with idiopathic tinnitus, including their psychological status, are explored. It also has great positive significance for the dialectic and treatment of Chinese medicine.

RETRACTED

The results of this study showed that the average age and the longest course of the disease were the oldest and the longest in the kidney essence depletion group among all syndrome groups, while the wind-infested group had the shortest course of disease. Zhang Jingyue recorded in the “Jingyue Quanshu”: “The ear is the kidney orifice, where the ancestral veins gather… After middle age, every tinnitus… is due to yin failure and kidney deficiency.” It shows that virtual tinnitus caused by the loss of kidney essence is the most common and is closely related to age. The older you are, the more likely it is that the kidneys are weak, the ears are not prosperous, and the orifices are lost [13, 14]. The wind-evil invasion disease is a positive manifestation of exogenous feelings. At the same time, most of the patients have not decayed righteousness, have a rapid onset, rapid progress, and easy self-healing, so the course of the disease is relatively short.

Traditional Chinese medicine has always paid attention to the role of emotional factors in the occurrence and development of diseases. “Su Wen” records: “The heart hides the mind, the lungs hide the soul, the liver hides the soul, the spleen hides the meaning, and the kidney hides the will.” It shows that various mental activities will have an impact on the corresponding viscera [15]. In this study, patients with all syndromes have sleep disorders, In addition, the anxiety of patients in the phlegm-fire stagnation and liver-fire disturbance group was more severe than that in the spleen and stomach weakness and kidney essence loss group, while the depression of the spleen-stomach weakened and kidney essence-deficient group patients was heavier than that in the spleen-fire stagnation and liver-fire disturbance group. The possible causes are phlegm-fire stagnation and liver-fire disturbance, which are empirical tinnitus, and the course of the disease is relatively short. The patient pays more attention to tinnitus, has poor adaptability, and is prone to anxiety. However, the weak spleen and stomach and the loss of kidney essence belong to the deficient tinnitus, and the course of the disease is relatively short. Long, patients are often forced to adapt and are not prone to anxiety, but this can cause long-term sleep disturbances, produce bad moods, and make them more prone to depression [16, 17].

RETRACTED

Idiopathic tinnitus may be with or without hearing loss. A survey conducted by Zhang and Zhang [18] on 2171 cases of tinnitus patients showed that, about 75.29% of tinnitus patients had hearing loss, mainly mild to moderate. In this study, the kidney essence loss group has the highest total hearing loss rate among all syndrome groups, and high-frequency and mild hearing losses are the main ones. The total hearing loss rate of the wind evil invasion group was the lowest. It is suggested that, in addition to being the most common in all tinnitus patients, patients with kidney essence loss often have premature cochlear aging, but when their hearing impairment has not yet developed to the language frequency, the patient still does not know it and requires physicians to clinically intervene as soon as possible. Hearing loss in the high-frequency area is a microscopic syndrome differentiation index for patients with kidney essence loss, which has certain significance. Because of the shorter course of disease and better physiological functions in patients with wind pathogen invasion, they are often not accompanied by hearing loss [19, 20].

Earlier empirical tinnitus is mostly described by low-medium-frequency sounds such as “Weng Weng sound” and “whooping sound,” while virtual tinnitus is usually described by low-medium frequency sounds such as “cicada chirping” and “squeaking sound.” In addition, “Jingyue Quanshu” also has recorded “If the patients often heard the louder noise, it indicates the syndrome of excess,… if the patients often heard the small volume of noise, it indicates the syndrome of deficiency [21].” In this study, the tinnitus low-medium-frequency tone matching rate and tinnitus loudness in the wind pathogen invasion, liver-fire disturbance, and phlegm-fire stagnation group were higher than those in the spleen and stomach weakness and kidney essence loss group. The matching rate of high-frequency tones is lower than that of the weak spleen and stomach group and the kidney essence loss group, which is consistent with the above views. There was no obvious difference in the severity of tinnitus among the groups, with mild and moderate tinnitus being the main ones.

In summary, the clinical characteristics and psychoacoustic indexes of patients with idiopathic tinnitus are related to the TCM syndrome types. Patients with kidney-deficiency tinnitus tend to be older, have a longer course of disease, and are often accompanied by mild hearing loss in high-frequency areas. The course of disease is often shorter in patients with wind pathogen invasion. Positive tinnitus tends to have lower tinnitus tone than deficiency tinnitus and louder than deficiency tinnitus. In addition, all tinnitus patients have sleep disorders, and most tinnitus patients may have different degrees of psychological disorders except for the invasion of wind pathogens. This suggests that, in the treatment of idiopathic tinnitus, in addition to the disease itself, we should pay more attention to the patient's psychological condition. Combining psychotherapy could be regarded as a treatment method to obtain the best curative effect. This study revealed the differences in clinical characteristics of tinnitus patients with different TCM syndrome types and revealed the internal relationship between tinnitus and patients' psychological emotions, which provided a good reference value for TCM syndrome differentiation and treatment. However, there are still some shortcomings, such as too few samples, the differences in clinical characteristics between different syndrome types and the specific mechanism of the close relationship between tinnitus and psychological factors, which need to be further studied.

RETRACTED

## Figures and Tables

**Figure 1:** Sleep quality, anxiety, and depression scores of patients with different syndrome types (*n*, $\bar{x}$ ± *s*, points). The data were calculated as mean ± S.D. An asterisk (^*∗*^) indicates significant difference (*P* < 0.05) by *t*-test.

**Table 1:** Comparison of general conditions of patients with various syndrome types (*n*, %).

Group	Gender		Age (year)	Course of disease (months)	Side	
	Male	Female			Unilateral	Bilateral
Wind evil invasion group (*n* = 61)	32	29	41.42 ± 13.65^b^	1.14 ± 0.42	51	10
The liver fire disturbance group (*n* = 69)	37	32	45.98 ± 10.78^b^	3.73 ± 1.11^ab^	52	17
Phlegm-fire stagnation group (*n* = 42)	19	23	42.63 ± 11.57^b^	3.65 ± 1.34^ab^	35	7
Spleen and stomach weakness group (*n* = 48)	24	24	49.62 ± 9.87^b^	4.19 ± 1.08^ab^	38	10
Kidney essence loss group (*n* = 92)	51	41	60.32 ± 7.63	12.83 ± 5.76^a^	69	23
*F*/*χ*^2^ value	0.600		5.324	5.793	0.904	
*P* value	0.439		0.026	0.021	0.341	

Note: compared with the wind evil invasion group, ^a^*P* < 0.05; compared with the kidney essence loss group, ^b^*P* < 0.05.

**Table 2:** Comparison of average hearing threshold and hearing loss of patients with different syndrome types (*n*, %).

Group	Low frequency			High frequency			Completeness of hearing	Total hearing loss rate
	Mild	Moderate	Severe	Mild	Moderate	Severe		
Wind evil invasion group (*n* = 61)	1	1	0	2	1	0	56	5 (8.19)
The liver fire disturbance group (*n* = 69)	4	2	2	9	7	3	42	27 (39.13)^ab^
Phlegm-fire stagnation group (*n* = 42)	2	4	1	5	6	0	24	18 (42.86)^ab^
Spleen and stomach weakness group (*n* = 48)	1	3	1	9	2	4	34	20 (41.67)^ab^
Kidney essence loss group (*n* = 92)	12	9	4	39	15	6	7	85 (92.39)^a^
*χ*^2^ value								4.531
*P* value								0.032

Note: compared with the wind evil invasion group, ^a^*P* < 0.05; compared with the kidney essence loss group, ^b^*P* < 0.05.

RETRACTED

**Table 3:** Comparison of tinnitus in patients with different syndrome types (*n*, ±*s*).

Group	Tinnitus tone			Tinnitus loudness (dBHL)	THI score				
	Medium and low frequency	High frequency	No match frequency		Grade 1	Grade 2	Grade 3	Grade 4	Grade 5
Wind evil invasion group (*n* = 61)	47^ab^	9^ab^	5	4.32 ± 1.13^ab^	9	24	17	6	5
The liver fire disturbance group (*n* = 69)	57^ab^	7^ab^	5	9.72 ± 1.34^ab^	10	23	26	6	4
Phlegm-fire stagnation group (*n* = 42)	31^ab^	7^ab^	4	7.56 ± 2.46^ab^	5	18	12	4	3
Spleen and stomach weakness group (*n* = 48)	5	40	3	3.19 ± 1.07	6	23	12	4	3
Kidney essence loss group (*n* = 92)	11	79	2	2.88 ± 0.96	3	37	48	2	2
*F*/*χ*^2^ value	8.271			2.967	3.956				
*P* value	0.008			0.034	0.123				

Note: compared with the weak spleen and stomach group, ^a^*P* < 0.05; compared with the kidney essence loss group, ^b^*P* < 0.05.

## Data Availability

The data used during the study are available from the corresponding author upon request.
